The article "The Clinical Diagnostic Value of F-FDG PET/CT Combined with MRI in Pancreatic Cancer" was published in 2022. Journal: Contrast Media Mol Imaging.

# The Clinical Diagnostic Value of F-FDG PET/CT Combined with MRI in Pancreatic Cancer

**DOI:** 10.1155/2022/1479416

**Published:** 2022-08-04

**Authors:** Xinyan Liu, Yi Ren, Jianying Wang, Xiujin Yang, Li Lu

**Affiliations:** Chongqing Universal Hongling Medical Imaging Diagnostic Center, Yuzhong, Chongqing 400000, China

## Abstract

Pancreatic cancer is a common gastrointestinal tumor with increasing morbidity and mortality, and it is difficult to differentiate it from chronic mass pancreatitis. F-18-fluorodeoxyglucose positron emission tomography/computed tomography (F-FDG PET/CT) can be used for diagnosis of pancreatic cancer, staging, radiotherapy planning, evaluation of efficacy and recurrence, and differentiation from posttreatment fibrosis but the sensitivity and specificity of diagnosis of chronic pancreatitis are poor. Magnetic resonance imaging (MRI) not only shows the morphology, location, and size of organs and lesions but also has the advantages of low radiation, high soft tissue contrast, and multiparameter imaging, which can help determine the nature of occupying pancreatic lesions. In this study, the watershed algorithm (WA) was used to segment the abdominal images to extract images of pancreatic cancer cells and to compare the value of F-FDG PET/CT combined with MRI in the diagnosis of pancreatic occupying lesions.

## 1. Introduction

Pancreatic cancer is the most common type of malignant tumor [1, 2], and according to the World Health Organization 2021 statistics, 9.7 million people die of pancreatic cancer worldwide each year, and pancreatic cancer has become an important threat to human life and health [3]. The early stage of pancreatic cancer is usually asymptomatic, and medical statistics show that 80% of pancreatic cancer patients are diagnosed at an advanced stage, thus losing the best time for treatment [4, 5]. However, current medical clinical practice shows that one-third of pancreatic cancer is potentially curable if early diagnosis and early treatment are achieved, so the treatment of pancreatic cancer is very dependent on its early diagnosis [6]. Because the pancreatic blood flow is rich, and the pathological bleeding risk of routine puncture biopsy is high, the pancreatic tumor can be preliminarily diagnosed clinically in combination with the patient's symptoms and auxiliary examinations, and the pathological examination can be improved and further confirmed at the same time of surgical treatment. Clinical symptoms such as obstructive jaundice, progressive exacerbation of jaundice, abdominal distension and pain, anorexia, weight loss, fixed abdominal mass, ascites, and even distant metastasis. Auxiliary examinations include serum CEA, CA199, B-ultrasound, CT, MRI, ERCP, etc.

The article "The Clinical Diagnostic Value of F-FDG PET/CT Combined with MRI in Pancreatic Cancer" was published in 2022. Journal: Contrast Media Mol Imaging.

In addition, with the continuous improvement of the social and economic level, the concept of “early detection and treatment of diseases” is becoming more and more recognized, which also puts more demands on disease diagnosis techniques [7]. In the clinical diagnosis of medicine, only pathological examination can be used as a means of confirming the diagnosis, and pathological examination is the “gold standard” for pancreatic cancer diagnosis, which is often a qualitative diagnosis made by the doctor through microscopic observation of the pathological characteristics of the cells, combined with the doctor's diagnostic experience and professional knowledge. By observing the pathological section under high magnification, the pathologist will check whether there are specific cells in the section and statistically analyze their number, distribution, morphology, and other characteristics. A large number of cells in each field of view and the need to observe dozens or hundreds of fields of view in a single pathology section led to such a traditional approach that is not only subjective and prone to misdiagnosis but also requires a lot of time and effort on the part of the physician. The rapid development of computer technology and image processing technology has made it possible to apply computer-aided diagnosis technology in clinical practice more efficiently. In the clinical practice of pancreatic cancer diagnosis, the use of computer-aided diagnosis technology can help doctors to quickly detect and segment tumor cells, and on the basis of this, statistics and analysis can be performed, which can provide supplementary reference for doctors' diagnosis [8]. In clinical diagnostic practice, extraction of regions of interest from cell images is a key step, which is usually circled by physicians manually. The subsequent image feature extraction and analysis directly depend on the merit of the segmentation results, which ultimately affects the doctor's diagnosis. Introducing medical image segmentation techniques, it can help physicians to achieve the extraction of regions of interest from images [9]. Medical image segmentation mainly deals with the segmentation of various images involved in the medical field such as the common magnetic resonance (MRI) scanning images. Its main task is to segment regions of interest from these medical images such as specific organ parts, interest targets (such as tumors), and so on.

With the widespread use of F-18-fluorodeoxyglucose positron emission tomography/computed tomography (F-FDG PET/CT) in oncology, pancreatic F-FDG PET/CT provides clinicians, especially surgeons, with a qualitative diagnosis of the disease, the preoperative assessment of pancreatic occupancy, postoperative monitoring and other information, which increases the assurance of choosing an effective and efficient treatment plan for patients [10–12]. Pancreatic cancer can ingest a large amount of 18F-FDG. On 18F-FDG PET/CT, it shows abnormal radioactive concentration at the pancreatic tumor site, that is, hypermetabolic lesions. A single injection of 18F-FDG can be used for whole-body imaging. Therefore, PET whole-body imaging can not only detect the primary tumor at an early stage but also comprehensively understand the whole-body involvement range of the disease, providing an objective basis for the accurate staging and selection of appropriate treatment schemes in clinical practice. The limitations of the current studies reported on the application of pancreatic F-FDG PET/CT include a limited sample size in a single center; comparative studies mainly with CT imaging; and the qualitative diagnosis confirmed by follow-up in some cases without a pathological basis. This study retrospectively analyzed patients with pancreatic lesions, all of whom underwent F-FDG PET/CT and Magnetic resonance imaging (MRI), and all of whom had a clear pathological diagnosis by surgery or puncture, which can provide some clinical reference experience of F-FDG PET/CT imaging. This paper is divided into the following five sections: Section 1 briefly introduces the research background and main structure of this paper; Section 2 introduces the current domestic and international research and the significance of this paper; Section 3 introduces the abdominal image segmentation scheme based on watershed algorithm (WA); Section 4 investigates the effect of F-FDG PET/CT combined with MRI on pancreatic cancer and the clinical diagnostic value of F-FDG PET/CT combined with MRI for pancreatic cancer; and Section 5 summarizes the research content and future research directions of this paper.

The article "The Clinical Diagnostic Value of F-FDG PET/CT Combined with MRI in Pancreatic Cancer" was published in 2022. Journal: Contrast Media Mol Imaging.

## 2. Related Works

The high 5-year mortality rate and poor prognosis of patients with pancreatic cancer are the focus of clinical oncology research. In pancreatic cancer, early detection and surgical resection is the only treatment that offers a chance of cure. The National Comprehensive Cancer Network (NCCN) guidelines recommend the use of pancreatic CT or MRI, chest imaging, and ultrasound endoscopy to determine the resectability of pancreatic cancer. However, the NCCN does not recommend PET/CT as a staging test, noting that its role remains unclear due to the lack of data on the clinical use of validated PET/CT scans. Pancreatic cancer studies have shown an overall sensitivity of 92% for PET scans alone. Studies have also shown that PET/CT has the potential to guide the management of patients with pancreatic cancer, and in some cases, it may be more beneficial than imaging with CT or MRI but its tests are expensive.

To date, the etiology of pancreatic cancer is unknown, and known risk factors include smoking, obesity, genetics, diabetes, diet, and physical inactivity [13, 14]. Studies also show that elderly patients are common; the prevalence of males is higher than that of females; long-term exposure to toxic chemicals, such as long-term exposure to n-nitrosomethylamine, alkylates and other chemicals will increase the risk of pancreatic cancer; patients with chronic pancreatitis have a correspondingly higher risk of developing pancreatic cancer; and African Americans are more likely to develop pancreas than the whites. Despite the low 5-year survival rate after surgical resection of pancreatic cancer patients, surgery remains the cornerstone of treatment for patients with resectable pancreatic tumors. In patients with this fatal cancer, assessing the accurate staging and resectability of the tumor is crucial to determine the most appropriate treatment option (e.g., surgical resection, postsurgical neoadjuvant therapy, or palliative care) and to predict the patient's prognosis [15]. It has been shown that F-FDG PET/CT can reveal pancreatic and extrapancreatic lesions in patients with pancreatic cancer, providing more specific information for the diagnosis and understanding of the pathological features of pancreatic cancer [16]. F-FDG PET/CT can be used for diagnosis, early staging, treatment response assessment, differentiation of recurrent tumors from posttreatment fibrosis, and radiation treatment planning [17]. In addition, due to the increasing proportion of patients initially considered surgical candidates, F-FDG PET/CT may be a cost-effective way to identify patients with a true surgical indication [18]. However, the prognostic value of F-FDG PET/CT in patients with pancreatic cancer is controversial, and there is no consensus on its predictive ability.

In addition, with the rapid development of computer technology and image processing technology, computer-aided diagnosis technology can be more effectively applied in clinical practice. In the clinical practice of cancer diagnosis, the use of computer-aided diagnosis technology can help doctors to quickly detect and segment tumor cells, and on the basis of this, perform statistics and analysis, thus providing doctors with supplementary references for diagnosis. In clinical diagnostic practice, extraction of regions of interest from cell images is a key step, which is usually circled by physicians manually [19]. The subsequent image feature extraction and analysis directly depend on the merit of the segmentation results, which ultimately affects the physician's diagnosis. Introducing medical image segmentation techniques, it can help physicians to achieve the extraction of regions of interest in images.

The article "The Clinical Diagnostic Value of F-FDG PET/CT Combined with MRI in Pancreatic Cancer" was published in 2022. Journal: Contrast Media Mol Imaging.

Without the help of computer-aided diagnostic techniques, the work of pathologists in reading films would be intense and inefficient, and there is also a certain amount of personal subjectivity in manual recognition, which makes the recognition accuracy vary from doctor to doctor [20]. Therefore, it is necessary to study how to detect and recognize cell images efficiently and accurately, which will help physicians to complete the intense work of reading films faster and better. Image segmentation is the cutting of an image into different sub-regions, each of which is specific in its own nature, and the rules of cutting depend on the problem to be solved. The main applications of image segmentation include the following: (1) medical image analysis; (2) military research field; (3) remote sensing meteorological service; (4) traffic image analysis; and (5) object-oriented image compression and content-based image database query. WA is a powerful method for image segmentation, which can better extract the regions of interest in the image for study. Many existing studies have shown that WA is an effective image segmentation method but it usually needs to be used in combination with other methods in order to obtain better segmentation results. How to combine WA with other methods for effective use is the problem that needs to be studied in this paper. An important idea to improve WA is to use prior knowledge. It would greatly increase the efficiency of segmentation and mitigate oversegmentation if possible, target regions are marked before performing watershed segmentation.

In view of this, this study extracted abdominal images by WA and comprehensively investigated the effects of F-FDG PET/CT and MRI on staging, vascular invasion, distant metastasis, and surgical indications in pancreatic cancer patients.

## 3. Watershed Algorithm-Based Abdominal Image Cutting Scheme

After H&E staining, the cell nuclei will be stained blue-purple by hematoxylin, and most of the cell nuclei have a circular outline, and the circle has a good radial symmetry property, so this paper achieves the detection of the center of the cell nuclei by fast radial symmetry transformation and uses the center coordinates as foreground markers, so as to achieve the watershed segmentation based on foreground markers for the cell images. The image segmentation algorithm and process used in this paper can be described as follows: firstly, the principal component extraction, the H-staining component map of the H&E-stained pancreatic cancer cell image, i.e., the grayscale map of the hematoxylin part, is extracted by the color deconvolution technique; then the image preprocessing is applied to this grayscale map by morphological methods and image denoising techniques; then the cell center coordinates are obtained by the fast radial symmetric transform and used as the foreground Then, the cell center coordinates are obtained by fast radial symmetric transformation and used as foreground markers; finally, the foreground markers are combined with the watershed algorithm to achieve cell segmentation. The flow chart of the improved watershed algorithm based on foreground markers is shown in Figure 1.

The article "The Clinical Diagnostic Value of F-FDG PET/CT Combined with MRI in Pancreatic Cancer" was published in 2022. Journal: Contrast Media Mol Imaging.

The H&E staining method, known as hematoxylin-eosin staining, takes advantage of the fact that different components of the cells have different affinities for hematoxylin and different staining properties, and after hematoxylin staining, the cell nuclei, etc., are blue. Using this property, the hematoxylin staining part needs to be extracted separately, i.e., the main component extraction.

After H&E staining, the nuclei of pancreatic cancer cells will be stained purple by hematoxylin, so the grayscale map of the hematoxylin-stained part needs to be extracted, and all subsequent steps will be performed on that grayscale map. Color separation and quantitative analysis of H&E-stained color images can be performed using the color deconvolution technique. By performing color deconvolution on RGB images, the contribution of each stain can be calculated based on the absorbance of the particular stain. The optical density of each channel in the RGB color space can be defined as

(1) $$\begin{array}{c} OD_{C}=-\log_{10}\left(\frac{I_{C}}{I_{0,C}}\right),\\ =A^{*}C_{c}, \end{array}$$

where *I*_0,*c*_ is the incident light, *I*_*C*_ is the outgoing light, A is the amount of dye action, and *C*_*c*_ is the light absorption factor. From equation (1), the value of *O*  *D* for each channel is linearly related to the concentration of the absorbing material. A vector of 3 × 1 can be used to represent the optical density value of each dye for each channel in RGB, so the color system using 3 dyes can be expressed as

(2) $$\begin{array}{c} \left[\begin{array}{ccc} p_{11} & p_{12} & p_{13}\\ p_{21} & p_{22} & p_{23}\\ p_{31} & p_{32} & p_{33} \end{array}\right], \end{array}$$

where the rows correspond to each stain and the columns correspond to the optical density of each strain under the *R*, *G*, and *B* channels, respectively, we can call this matrix the OD matrix. By measuring the relative absorbance of red, green, and blue on slides stained with a single stain, the staining specificity value of OD for each of the three channels can be easily determined.

The article "The Clinical Diagnostic Value of F-FDG PET/CT Combined with MRI in Pancreatic Cancer" was published in 2022. Journal: Contrast Media Mol Imaging.

In order to separate the different colorings, an orthogonal transformation of the RGB information is required to obtain the contribution of each coloring. The following are the steps of color deconvolution.

### 3.1. Normalized  OD Matrix

For each component of the OD vector divide the length of the vector, e.g., equations (2)–(4):

(3) $$\begin{array}{c} {\hat{p}}_{11}=\frac{p_{11}}{\sqrt{p_{11}^{2}+p_{12}^{2}+p_{13}^{2}}}, \end{array}$$

(4) $$\begin{array}{c} {\hat{p}}_{21}=\frac{p_{21}}{\sqrt{p_{21}^{2}+p_{22}^{2}+p_{23}^{2}}}, \end{array}$$

(5) $$\begin{array}{c} {\hat{p}}_{31}=\frac{p_{31}}{\sqrt{p_{31}^{2}+p_{32}^{2}+p_{33}^{2}}}. \end{array}$$

### 3.2. Deconvolution

Let *C* be the vector of 3 × 1, representing the contribution of each dye on each pixel (assuming the number of stains is 3), then the OD value of the point in OD space is *y*=*CM*, obviously, the inverse matrix of the required *C*=*M*^−1^[*y*], OD matrix is the color deconvolution matrix *D*=*M*^−1^, so the orthogonalized image is represented as

(6) $$\begin{array}{c} C=D\left[y\right]. \end{array}$$

For hematoxylin, eosin, and DAB, the matrix *D* is

(7) $$\begin{array}{c} \begin{array}{ccc} 1.88 & -0.07 & -0.60\\ -1.02 & 1.13 & -0.48\\ -0.55 & -0.13 & 1.57 \end{array}. \end{array}$$

Some noise may be generated when the pathological slides are made into cell images by the scanner; also the cell images may be contaminated by external noise during transmission. Therefore, it is necessary to filter and denoise the cell images. Most of the image noise belongs to Gaussian noise, so Gaussian filtering is widely used in the field of image noise reduction. The two-dimensional Gaussian distribution is

(8) $$\begin{array}{c} G\left(x,y\right)=\frac{1}{\sqrt{2\pi }\sigma^{2}}e^{-x^{2}+y^{2}/2\sigma^{2}}. \end{array}$$

After Gaussian filtering, the noise of the image is suppressed, but at the same time the image is blurred, so in order to keep the image edge information clear, it is necessary to perform bilateral filtering again. Bilateral filtering is a kind of nonlinear filter, which can make the edges of the image smoother.

Equations (10) and (11) give the operation of bilateral filtering, *I*_*q*_ is the input image, and *I*_*p*_^*bf*^ is the filtered image:

(9) $$\begin{array}{c} I_{P}^{bf}=\frac{1}{W_{P}^{bf}}\sum_{q\in S}G_{\sigma_{s}}\left(\left\|p-q\right\|\right)G_{\sigma_{r}}\left(\left|I_{p}-I_{q}\right|\right)I_{q}. \end{array}$$

Among them,

(10) $$\begin{array}{c} W_{P}^{bf}=\sum_{q\in S}G_{\sigma_{s}}\left(\left\|p-q\right\|\right)G_{\sigma_{r}}\left(\left|I_{p}-I_{q}\right|\right). \end{array}$$

Even after the filtering and denoising operation, the cell images often have some cluttered structures. At this point, the purpose of removing these structures can be achieved by using only some morphological grayscale reconstruction. By performing morphological open reconstruction, those bright targets that are smaller than the structural elements will be removed. Similarly, by performing morphological closed reconstruction, dark targets that are smaller than the structural elements will be removed. By alternating these two operations, a smoother image is produced. In addition, the size of the structural elements can be adjusted to fit the needs. Here the morphological open reconstruction is performed first, followed by the morphological closed reconstruction. Of course, the selection of the size of the structural elements is based on a combination of the size of the cell nucleus and the filtered structures, and the image resolution.

The article "The Clinical Diagnostic Value of F-FDG PET/CT Combined with MRI in Pancreatic Cancer" was published in 2022. Journal: Contrast Media Mol Imaging.

While the previously mentioned morphological transformations involve only one image and one structural element, geodesic expansion involves two images: a marker image and a mask image. Its basic idea is to perform the expansion operation on the marker image with a specific structure element and to restrict the resulting image with the mask image.

Let *f* be the marker image, *g* be the mask image, and the geodesic expansion of *f* to *g* be *δ*_*g*_(*f*), which is defined as the point-by-point minima between the mask image and the expanded image, as shown in the following equation:

(11) $$\begin{array}{c} \delta_{g}\left(f\right)=\delta \left(f\right)\wedge g. \end{array}$$

Geodesic *ε*_*g*_(*f*) erosion is the dyadic operation of geodesic expansion, and the geodesic expansion of *f* to *g* is defined as the point-by-point maximum between the mask image and the expansion image, i.e.,

(12) $$\begin{array}{c} \varepsilon_{g}\left(f\right)=\varepsilon \left(f\right)\wedge g. \end{array}$$

From the definition of geodesic expansion and geodesic erosion, it can be seen that the geodesic transformation is applied to the image several times, and after a certain number of times, the expansion or contraction of the image will be completely prevented by the masked image. This indicates that multiple geodesic transformations will result in a stable resultant image.

Denote the expansion reconstruction of *f* to *g* as *R*_*g*_^*δ*^(*f*), which is defined as the geodesic expansion cycle of *f* to *g* until the resultant image is stable, as shown in the following equation:

(13) $$\begin{array}{c} R_{g}^{\delta }\left(f\right)=\delta_{g}^{\left(i\right)}\left(f\right), \end{array}$$

where *i* denotes the number of cycles when the result is stable.

The article "The Clinical Diagnostic Value of F-FDG PET/CT Combined with MRI in Pancreatic Cancer" was published in 2022. Journal: Contrast Media Mol Imaging.

The corrosion reconstruction of *f* on *g* is *R*_*R*_^*ε*^(*f*), which is defined as the geodesic corrosion cycle of *f* on *g* until the resultant image is stable, as shown in the following equation:

(14) $$\begin{array}{c} R_{g}^{\varepsilon }\left(f\right)=\varepsilon_{g}^{\left(t\right)}\left(f\right), \end{array}$$

where *i* denotes the number of 㵌-loops when the result is stable.

The open reconstruction of the image *f* is a reconstruction of the corrupted image of *f*, as shown in the following equation:

(15) $$\begin{array}{c} \gamma_{R}\left(f\right)=R_{f}^{\delta }\left[\varepsilon \left(f\right)\right]. \end{array}$$

The open reconstruction keeps the components of the image that are not corrupted. The pairwise operation of open reconstruction during closed reconstruction is shown in the following equation:

(16) $$\begin{array}{c} \varphi_{R}\left(f\right)=R_{f}^{\varepsilon }\left[\delta \left(f\right)\right]. \end{array}$$

After the open and closed reconstructions, the nucleus outline usually has burrs and appears irregular. In this case, a smaller structural element is used for the closed operation to eliminate the burr and remove the excess adhesions, and simplify the target shape. The size of the structural element is half the size of the structural elements of the previous two operations.

The selection of structure elements is not a panacea but should be selected according to the actual situation, only slightly larger than the structure you want to filter out. If the structure element is selected too large, the detailed information of the image will not be obtained; and if the structure element is selected too small, the effect of filtering these structures will not be achieved, which will have a negative impact on the segmentation effect.

## 4. Diagnostic Analysis of Pancreatic Cancer by F-FDG PET/CT and MRI

According to the clinical treatment records, medical records, serological tumor marker test results, imaging data, and surgical records, it was found that among 101 patients with pancreatic cancer, 69 cases were diagnosed through clear case information, including 60 cases of pancreatic ductal cell carcinoma, 7 cases of mucinous cyst adenocarcinoma and 2 cases of medullary carcinoma; the remaining 32 cases were diagnosed through comprehensive clinical data and follow-up data. The tumor sites: 59 cases were located in the head of the pancreas and the leptomeningeal region, and 42 cases were located in the tail of the pancreatic body. 18F-FDG PET/CT results showed that 101 lesions were found in 101 patients, T1-2 in 35 cases, T3 in 32 cases, T4 in 34 cases, N1 in 45 cases, and M1 in 38 cases; MRI results showed that 93 lesions were found in 101 patients, T1-2 in 33 cases, T3 in 31 cases, T4 in 29 cases, and N1 in 42 cases. The tumor staging detection rate of MRI was 92.1%, which was lower than that of F-FDG PET/CT (100.0%) (*P* < 0.05), and the results are shown in Figure 2.

The article "The Clinical Diagnostic Value of F-FDG PET/CT Combined with MRI in Pancreatic Cancer" was published in 2022. Journal: Contrast Media Mol Imaging.

The staging results of pancreatic cancer showed that F-FDG PET/CT showed 35 cases of T1-2, 32 cases of T3, 34 cases of T4; 45 cases of N1, and 38 cases of M1; MRI results showed that 93 lesions were found in 101 patients, 33 cases of T1-2, 31 cases of T3, 29 cases of T4; 42 cases of N1 and 26 cases of M1. It can be seen that the tumor detection rate of MRI is lower than that of 18F-FDG PET/CT (*P* < 0.05), and the reasons for the missed diagnosis are: small lesions, insignificant density changes, or too small short diameter of lymph nodes, which may be due to the deep location of the pancreas, covered by the stomach and intestinal tissues, some pancreatic cancer lesions do not have significant density changes, and in more cases, pancreatic cancer lacks blood supply, so MRI and other detection methods are less sensitive and accurate for its The sensitivity and accuracy of MRI are not good, but its efficacy in assessing vascular invasion is better.

Vascular invasion was present preoperatively in 18 patients, of which 3 were confirmed by surgery and 15 by follow-up; distant metastases were present preoperatively in 54 patients, of which 16 were confirmed by surgery and 38 by follow-up; in the other 47 patients, no distant metastases were found and were confirmed by surgery and follow-up.18 The comparative results of F-FDG PET/CT and MRI for the assessment of vascular invasion and distant metastases in pancreatic cancer are shown in Figures 3–5. The difference was statistically significant (*P* < 0.05). F-FDG PET/CT was more effective in assessing distant metastases and MRI was more effective in assessing vascular invasion. The combination of the two methods was more effective in assessing vascular invasion and distant metastases than the single method.

As shown in Figure 3, the efficacy of the combination of both F-FDG PET/CT and MRI for the assessment of vascular invasion, distant metastases and surgical indications was better than that of the single method, with statistically significant differences (*P* < 0.05). The reason for this is that the multimodal imaging of glucose metabolism function imaging by F-FDG PET and anatomical structure imaging by CT is used to comprehensively evaluate the lesions, and it is a whole-body imaging, so it has a higher evaluation efficacy on the metabolic activity of tumor lesions and the sensitivity of pancreatic cancer diagnosis, which is consistent with the results of previous studies.

The article "The Clinical Diagnostic Value of F-FDG PET/CT Combined with MRI in Pancreatic Cancer" was published in 2022. Journal: Contrast Media Mol Imaging.

Thirty-five patients were confirmed to have surgical indications; 37 patients were confirmed to have no surgical indications, including 13 with vascular factors, 15 with metastatic factors, 6 with vascular combined with metastatic factors, and 3 with extensive adhesions that could not be completely resected and therefore palliative surgery was performed; 29 patients were confirmed to have no surgical indications at follow-up. The results of F-FDG PET/CT and MRI were statistically different (*P* < 0.05), and the results are shown in Figure 6. The combination of the two methods was more effective than the single method in assessing the indication for surgery.

MRI evaluation showed that 38 patients were not indicated for surgery, and surgery or follow-up confirmed that they were not indicated for surgery; enhanced CT evaluation showed that of the 63 patients with indications for surgery, 38 were confirmed as not indicated for surgery, and 18 of them were confirmed as not indicated for surgery by improving their clinical stage after F-FDG PET/CT verification, namely, one case of pulmonary metastasis, nine cases of liver metastasis, three cases of peritoneal 3 cases of metastasis, 2 cases of bone metastasis, and 3 cases of distant lymph node metastasis. There were still 20 cases that were misclassified as h0061ving an indication for surgery, as shown in Figure 7.

Analysis of the above data clearly shows the impact of F-FDG PET/CT combined with MRI on the treatment strategy, i.e., F-FDG PET/CT helps to better identify patients with a real surgical possibility in patients confirmed by MRI as having an indication for surgery. 38 of the 63 patients with an indication for surgery as shown by MRI evaluation were confirmed as having no indication for surgery, of which 18 Among them, 18 patients were confirmed as non-surgical after improvement of their clinical stage by F-FDG PET/CT verification: 1 with pulmonary metastasis, 9 with liver metastasis, 3 with peritoneal metastasis, 2 with bone metastasis, and 3 with distant lymph node metastasis. The MRI evaluation showed no indication for surgery in 38 cases, and no indication for surgery was confirmed by surgery or follow-up. It can be seen that F-FDG PET/CT is a whole-body scan, which can effectively compensate for the relatively limited scope of MRI, especially its accurate assessment of the M-stage, which led to the change of treatment plan for a significant number of patients. It is confirmed that F-FDG PET/CT helps to improve the detection of occult metastases, ultimately avoiding unnecessary surgery in these patients.

The article "The Clinical Diagnostic Value of F-FDG PET/CT Combined with MRI in Pancreatic Cancer" was published in 2022. Journal: Contrast Media Mol Imaging.

## 5. Summary and Outlook

Pancreatic cancer is the fourth most common cause of cancer-related death for both men and women in the United States. In the next 10 years, pancreatic cancer will become the second leading cause of cancer death after lung cancer. The purpose of this paper is to evaluate the efficacy of F-FDG PET/CT for the assessment of pancreatic cancer staging and resectability, and to detect occult metastatic disease in patients with resectable or borderline resectable pancreatic cancer to determine whether it can prevent ineffective open surgery. In this study, we found that among 101 patients with pancreatic cancer, 69 cases were diagnosed by definite pathological data, including 60 cases of pancreatic ductal cell carcinoma, 7 cases of mucinous cyst adenocarcinoma, and 2 cases of medullary carcinoma; the remaining 32 cases were diagnosed by comprehensive clinical data and follow-up data. According to the tumor site, 59 cases were located in the head of the pancreas and the leptomeningeal region, and 42 cases were located in the tail of the pancreatic body.

In summary, F-FDG PET/CT has better efficacy in assessing pancreatic cancer staging, distant metastases, and indications for surgery, and MRI has higher efficacy in assessing vascular invasion. f-FDG PET/CT can help improve the detection of occult metastases and can more accurately and effectively assist in the preoperative evaluation of patients. Researchers are currently working to identify biomarkers that will identify patients who may benefit from surgical treatment, and this will be the direction of subsequent studies, with the aim of providing a more complete plan for the diagnosis and treatment of pancreatic cancer patients through the collaboration of serology, imaging, pathology, and follow-up, in order to obtain more optimal treatment.

## Figures and Tables

**Figure 1:** Method flow chart.

**Figure 2:** Comparison of F-FDG PET/CT and MRI for TNM staging of pancreatic cancer.

**Figure 3:** Evaluation of vascular invasion and distant metastasis in pancreatic cancer by F-FDG PET/CT.

**Figure 4:** Evaluation of vascular invasion and distant metastasis in pancreatic cancer by MRI.

**Figure 5:** Evaluation of vascular invasion and distant metastasis in pancreatic cancer by F-FDG PET/CT and MRI.

**Figure 6:** Evaluation of vascular invasion and distant metastasis in pancreatic cancer by F-FDG PET/CT and MRI.

**Figure 7:** The flowchart of distributed neural optimization strategy for online routing green logistic systems.

## Data Availability

The figures used to support the findings of this study are included in the article.

The article "The Clinical Diagnostic Value of F-FDG PET/CT Combined with MRI in Pancreatic Cancer" was published in 2022. Journal: Contrast Media Mol Imaging.

## References

[1] Jegatheeson S., Dandrieux J. R. S., Cannon C. M. (2020). Suspected pancreatic carcinoma needle tract seeding in a cat. *Journal of Feline Medicine and Surgery Open Reports*.

[2] Guo J. Q., Yang Z. J., Wang S., Wu Z. Z., Yin L. L., Wang D. C. (2020). LncRNA SNHG16 functions as an oncogene by sponging miR200a3p in pancreatic cancer. *European Review for Medical and Pharmacological Sciences*.

[3] Kim J., Bassetti M. F., Raldow A. (2020). Focus on adaptive treatments for the first multi-institutional online adaptive radiation therapy trial (SMART) in pancreas cancer. *International Journal of Radiation Oncology, Biology, Physics*.

[4] Gits H. C., Tang A. H., Harmsen W. S. (2020). SMAD4 as a predictive biomarker for locally aggressive phenotype in resected pancreas cancer. *International Journal of Radiation Oncology, Biology, Physics*.

[5] Preston Hewgley W., Hester Caitlin A., Zeh Herbert J., Charles Yopp A., Marcelo Polanco P. (2020). Disparities in surgical resection for early stage pancreas cancer in the Texas-Mexico border population. *Journal of the American College of Surgeons*.

[6] Xiang M., Heestand G. M., Chang D. T., Pollom E. L. (2020). Neoadjuvant treatment strategies for resectable pancreas cancer: a propensity -matched analysis of the National Cancer Database. *Radiotherapy & Oncology*.

[7] Hecht E. M., Zins M., Tamm E. P. (2020). Editorial for “MRI vs. CT for the detection of liver metastases in patients with pancreatic carcinoma: a comparative diagnostic test accuracy systematic review and meta‐analysis”. *Journal of Magnetic Resonance Imaging*.

[8] Lin Q., Su L., Huang D., Song X., Liu J., Liu X. (2020). Pancreatectomy combined with arterial resection for pancreatic carcinoma with arterial infiltration: a meta-analysis. *Indian Journal of Surgery*.

[9] Ammarah G., Junaid Zia H., Abdul M., Hashmi Q. (2020). Chylous ascites a rare initial presentation of pancreatic carcinoma. *Journal of the College of Physicians and Surgeons Pakistan JCPSP*.

[10] Hui N. C., Zhang Y., Zhou G. (2020). Analysis of the efficacy of transcatheter arterial infusion chemotherapy in the treatment of pancreatic carcinoma. *Journal of Interventional Medicine*.

[11] Ali E. M., Maklad A. M., Khallaf S. M. (2020). Prolonged infusion of low dose gemcitabine in advanced pancreatic carcinoma. *Journal of Cancer Therapy*.

[12] Gouri P., Anuradha K., Singh A. (2021). A Comprehensive Review of the Multifaceted Role of the Microbiota in Human Pancreatic Carcinoma. *Seminars in cancer biology*.

[13] Heger U., Mack C., Hinz U., Hackert T., Büchler M. W., Strobel O. (2021). Surgical resection of isolated local recurrence in pancreatic carcinoma. *Pancreatology*.

The article "The Clinical Diagnostic Value of F-FDG PET/CT Combined with MRI in Pancreatic Cancer" was published in 2022. Journal: Contrast Media Mol Imaging.

[14] Horowitz D. P., Goodman K., Kachnic L. A. (2021). Ablative radiotherapy for patients with inoperable pancreas cancer-ready for prime time?. *JAMA Oncology*.

[15] Nehlsen A. D., Goodman K. A. (2021). Controversies in radiotherapy for pancreas cancer. *Journal of Surgical Oncology*.

[16] Hanada K., Fukuhara M., Minami T. (2021). Pathological features and imaging findings in pancreatic carcinoma in situ. *Pancreas*.

[17] Salahuddin M. K., Waheed Z., Muhammad A. J. (2021). Unusual presentation of metastatic pancreatic carcinoma. *Journal of the Pakistan Medical Association*.

[18] Khetan K., Baloda V., Sahoo R. K. (2019). SPARC expression in desmoplastic and non desmoplastic pancreatic carcinoma and cholangiocarcinoma. *Pathology, Research & Practice*.

[19] Patel Sameer H., Edwards Michael J., Ahmad Syed A. (2019). Intracellular ion channels in pancreas cancer.. Cellular physiology and biochemistry. *International Journal of Experimental Cellular Physiology, Biochemistry, and Pharmacology*.

[20] Fumitaka N., Takano Y., Kobayashi T. (2019). [Six cases of anaplastic pancreatic carcinoma diagnosed by endoscopic ultrasound-guided fine needle aspiration]. *Nihon Shokakibyo Gakkai zasshi = The Japanese journal of gastro-enterology*.

